The article "Sirtuin 6 contributes to migration and invasion of osteosarcoma cells via the ERK1/2/MMP9 pathway" was retracted in 2022. Reasons: duplicated images; signs of a paper mill; unreliable results or conclusions.

# Sirtuin 6 contributes to migration and invasion of osteosarcoma cells via the ERK1/2/MMP9 pathway

**DOI:** 10.1002/2211-5463.12265

**Published:** 2017-07-31

**Authors:** Hang Lin, Yi Hao, Zhengxu Zhao, Yongjun Tong

**Affiliations:** ^1^ Department of Orthopedics Zhejiang Hospital Hangzhou China

**Keywords:** ERK1/2, invasion, migration, MMP9, OS, SIRT6

## Abstract

Dysregulation of sirtuin 6 (SIRT6) is actively involved in tumor progression. High levels of SIRT6 have been associated with hepatocellular carcinoma and non‐small cell lung cancer, and SIRT6 facilitates growth and metastasis of cancer cells. However, the clinical significance and biological function of SIRT6 are not known for osteosarcoma (OS). Here, we report that SIRT6 was notably overexpressed in OS tissues compared with non‐cancerous specimens. The high level of SIRT6 was prominently correlated with malignant clinical parameters and poor prognosis of OS patients. SIRT6 was also up‐regulated in OS cells. SIRT6 knockdown inhibited the invasion and migration of Saos‐2 and U2OS cells *in vitro*, while SIRT6 restoration increased these cellular biological behaviors in MG‐63 cells. Mechanistically, SIRT6 up‐regulated expression of matrix metallopeptidase 9 (MMP9) in OS cells. MMP9 restoration partially abolished the effects of SIRT6 knockdown on OS cells, with increased cell migration and invasion. MMP9 knockdown reduced migration and invasion of SIRT6‐overexpressing MG‐63 cells. Furthermore, SIRT6 positively modulated the levels of phosphorylated extracellular signal‐regulated kinases 1 and 2 (ERK1/2). PD098059 and PD0325901, inhibitors of mitogen‐activated protein kinase kinase (MEK), blocked the regulatory effects of SIRT6 on p‐ERK1/2 and MMP9 levels, suggesting that SIRT6 regulated MMP9 abundance probably through the MEK–ERK1/2 pathway. These results suggest that SIRT6 may act as a prognostic predictor and a drug target for OS patients.

**Abbreviations**
ERK1/2: extracellular signal‐regulated kinases 1 and 2
HCC: hepatocellular carcinoma
MEK: mitogen‐activated protein kinase kinase
MMP9: matrix metallopeptidase 9
NSCLC: non‐small cell lung cancer
OS: osteosarcoma
SIRT6: sirtuin 6

Osteosarcoma (OS) is the commonest malignancies primarily initiated from bone and is usually presented in the metaphysis of long bones of children and young adults 1. Twenty‐ to 30‐year‐old young adults show the highest incidence of OS 2. Despite remarkable improvements having been achieved in treatment programs over the past decades, the prognosis of OS for children and adolescents remains poor 3. Therefore, it is important to discover a better molecular biomarker for predicting poor clinical response and prognosis of OS patients.

Sirtuin 6 (SIRT6), which belongs to the sirtuin family of NAD^+^‐dependent enzymes, has many pivotal functions and exhibits multiple enzymatic activities 4. There are three reported enzymatic activities of SIRT6: deacetylation, defatty‐acylation, and mono‐adenosine diphosphate (ADP) ribosylation 4. Recent studies have shown that SIRT6 functions as a tumor suppressor or oncogene in various human cancers 5, 6. Notably, SIRT6 overexpression induces apoptosis in tumor cells but not in normal cells 7. SIRT6 restrains proliferation via induction of apoptosis by repressing survivin in endometrial cancer 8. It is a key regulator of metabolism 5 and has been reported to down‐regulate gluconeogenesis in hepatocytes by enhancing GCN5‐mediated acetylation and inhibition of peroxisome proliferator‐activated receptor γ coactivator 1α 9. SIRT6 was shown to be a key regulator of fat homeostasis and obesity 10, which are associated with increased risk of several cancer types. Importantly, SIRT6 silencing results in tumor growth and glycolysis, suggesting that SIRT6 functions as a tumor suppressor by modulating cancer metabolism 11. Increased expression of SIRT6 prohibits the development of liver cancer by suppressing survivin 12 and correlates with a better clinical outcome in hepatocellular carcinoma (HCC) 13. Controversially, SIRT6 is reported to be overexpressed in HCC and its high expression is associated with malignant clinical features and shorter survival 14, 15. In addition, SIRT6 knockdown restrains growth of HCC *in vitro* and *in vivo* 14, 15. In pancreatic cancer, SIRT6 facilitates cancer cell migration by promoting Ca^2+^ responses 16, while Kugel *et al*. 17 showed that SIRT6 loss contributes to metastasis and progression of pancreatic ductal adenocarcinoma via modulation of Lin28b. Furthermore, SIRT6 is implicated in chemotherapy resistance and progression of breast cancer, and reduces the sensitivity of breast cancer to chemotherapeutic agents and then enhances cell proliferation and invasion 18, 19. SIRT6 functions as an oncogene and enhances cell proliferation and survival by promoting COX‐2 expression in skin cancer 20. In non‐small cell lung cancer (NSCLC), SIRT6 overexpression correlates with a poor prognosis and contributes to metastasis and chemotherapy resistance 21, 22. However, the clinical significance and biological role of SIRT6 in OS remain largely unknown.

In this study, we demonstrate that SIRT6 is overexpressed in OS tissues. OS patients with a high expression of SIRT6 show malignant clinical characteristics and reduced survival. Our results show that SIRT6 promotes migration and invasion of OS cells. Moreover, matrix metallopeptidase 9 (MMP9) is inversely regulated by SIRT6 and possibly functions in SIRT6‐induced migration and invasion of OS cells.

## Materials and methods

### Clinical samples

Sixty clinical specimens were obtained from patients who were histologically diagnosed as OS in the Department of Orthopedics, Zhejiang Hospital. Patients who received immunotherapy, chemotherapy or radiotherapy before surgical treatment were excluded. Informed consent was signed by each patient before clinical specimens were collected and used. All specimens were stored in liquid nitrogen for further investigation. The protocols involved for clinical specimens in this study were permitted by the Research Ethics Committee of Zhejiang Hospital.

### Cell culture and transfection

Human OS cell lines including U2OS, MG‐63, Saos‐2 and 143B were obtained from the American type culture collection (ATCC; Manassas, VA, USA). All cells were cultured in Dulbecco's modified Eagle's medium (DMEM; HyClone, Logan, UT, USA) along with fetal bovine serum (10%; HyClone) and antibiotics (Sigma‐Aldrich, St Louis, MO, USA). Cell cultures were kept in an incubator containing a 5% CO_2_ humidified atmosphere at 37 °C.

SIRT6 siRNA (siSIRT6; 5′‐CGAGGAUGUCGGUGAAUUA‐3′), SIRT6 and MMP9 overexpression plasmids (pcDNA3.1‐SIRT6 and pcDNA3.1‐MMP9), MMP9 siRNA (5′‐CAUCACCUAUUGGAUCCAATT‐3′) and corresponding control vectors were designed and synthesized by GenePharma (Shanghai, China). All vectors were then transfected into OS cells with Lippofectamine 2000 (Invitrogen, Carlsbad, CA, USA) following the manufacturer's protocol. Cells were exposed to 2′‐amino‐3′‐methoxyflavone (PD098059; 50 μm; Alexis, Bingham, UK) or PD0325901 (50 nm, Selleck Chemicals, TX, USA) for 30 min at 37 °C.

### Transwell assay and wound healing assay

Transwell chambers (Coring Costar, Cambridge, MA, USA) were employed to evaluate the migratory and invasive abilities of OS cells. OS cells were resuspended in serum‐free DMEM and subsequently seeded in the upper chambers. To induce the migration and invasion of OS cells, the lower chambers were filled with 600 μL DMEM supplemented with 20% fetal bovine serum. Forty‐eight hours after cell seeding, OS cells that migrated or invaded through the membranes (for invasion assay, the membranes were covered with 70 μL of Matrigel) were stained with crystal violet for cell counting under the microscope. A wound healing assay was conducted by using wound healing culture inserts (Ibidi, Munich, Germany) according to the manufacturer's instructions.

### Proliferation assay

For a 3‐(4,5‐dimethylthiazol‐2‐yl)‐2,5‐diphenyl‐tetrazolium bromide (MTT) assay, cells were seeded in 96‐well plates containing 100 μL DMEM per well. After transfection for 24, 48 and 72 h, 10 μL of MTT was added to each well and incubated for 4 h. Subsequently, 150 μL DMSO was added per well and a microplate reader (flexstation iii rom V2.1.28, Molecular Devices, Sunnyvale, CA, USA) was used to measure absorbance at 490 nm.

### Western blotting

Two days after transfection, total proteins were extracted and quantified with a BCA protein assay kit (Pierce, Bonn, Germany). Proteins were separated by 10% SDS/polyacrylamide gels and subsequently transferred to poly(vinylidene difluoride) membranes (Millipore, Bedford, MA, USA). After blocking with 5% non‐fat milk, the membranes were incubated with primary antibodies including SIRT6 (ab62739, Abcam, Cambridge, MA, USA), MMP9 (ab38898; Abcam), extracellular signal‐regulated kinases 1 and 2 (ERK1/2; ab17942; Abcam) and p‐ERK1/2 (no. 4370, Thr202/Tyr204; Cell Signaling Technology, Beverly, MA, USA). The secondary antibodies were obtained from Cell Signaling Technology (nos 7074 and 7076). α‐Tubulin (sc‐5286, Santa Cruz Biotechnology, Dallas, TX, USA) was used as a loading control. The protein bands on the membranes were detected with ECL Advance Western detection reagents (GE Healthcare, Little Chalfont, UK) and visualized with ChemiDoc XRS plus system (Bio‐Rad, Hercules, CA, USA).

### Statistical analysis

Data are presented as means ± SEM and analyzed by graphpad Prism 5 software (GraphPad Software, San Diego, CA, USA). The chi‐squared test was employed to explore the association between two variables. Student's *t* test and ANOVA were used to analyze continuous variable. Survival curves were constructed and differences between groups were analyzed using the Kaplan–Meier method and log‐rank test. A value of *P* < 0.05 was considered to be statistical significance.

## Results

### SIRT6 expression is up‐regulated in OS

To examine the expression status of SIRT6 in OS, immunoblotting was performed in 60 pairs of OS and corresponding non‐cancerous tissues. Our data disclosed that the levels of SIRT6 protein in OS tissues were increased compared with normal bone (NB) specimens (*P* < 0.05, Fig. 1A). Next, we compared the expressions of SIRT6 protein between OS cell lines and NB tissues. The levels of SIRT6 protein in all OS cell lines (U2OS, MG‐63, Saos‐2 and 143B) were significantly up‐regulated compared with NB tissues (*P* < 0.05 for all, Fig. 1B). These data indicate that SIRT6 probably plays an oncogenic role in OS.

**Figure 1:** The expression of SIRT6 in OS and NB tissues. (A) The altered expression of SIRT6 between OS tissues (*n* = 60) and adjacent NB specimens (*n* = 60). *P < 0.05. Numbers 1–6 refer to HCC tissues from case 1 to case 6. (B) The differences in the expression of SIRT6 between four different OS cell lines (Saos‐2, MG‐63, U2OS and 143B) and NB specimens. *P < 0.05.

### SIRT6 expression correlates with clinical parameters and prognosis of OS patients

To clarify the clinical significance of SIRT6 in OS, all patients were grouped into SIRT6 low group and SIRT6 high group according to the cut‐off value, which was defined as the median value of the cohort of patients tested. As shown in Table 1, OS patients expressing high SIRT6 had an advanced Enneking stage (*P* = 0.007), more metastasis (*P* = 0.010) and poor histological grade (*P* = 0.004). Furthermore, survival analyses indicated that OS patients expressing high SIRT6 showed a significantly reduced 5‐year overall survival and disease‐free survival (*P* = 0.033 and *P* = 0.028, respectively, Fig. 2A,B). We suggest that SIRT6 is a possible prognostic biomarker for OS patients.

**Table 1:** Correlation between the clinicopathological characteristics and SIRT6 expression in OS

Clinicopathological features	*n*	SIRT6 expression		*P*
		High	Low	
Gender				
Male	38	21	17	0.284
Female	22	9	13	
Age				
< 20	41	23	18	0.165
≥ 20	19	7	12	
Enneking stage				
I + IIA	38	14	24	0.007^a^
IIB + III	22	16	6	
Metastasis				
No	32	11	21	0.010^a^
Yes	28	19	9	
Histological classification				
Osteoblastic	35	16	19	0.432
Chondroblastic + Others	25	14	11	
Histological grade				
I + II	44	17	27	0.004^a^
III	16	13	3	

a Statistically significant.

**Figure 2:** The prognostic significance of SIRT6 in OS. All patients were grouped into SIRT6 low group (*n* = 30) and SIRT6 high group (*n* = 30) according to the cut‐off value, which was defined as the median value of the cohort of patients tested. Compared with SIRT6 low expression cases, SIRT6 high‐expression OS patients showed a significantly reduced (A) overall survival rate and (B) disease‐free survival rate.

### SIRT6 promotes the migration and invasion of OS cells

Tumor metastasis and recurrence are inseparable from enhanced cancer cell mobility 23. Thus, the functions of SIRT6 in modulating OS cell migration and invasion were further investigated. The expression of SIRT6 was knocked down by a specific siRNA in Saos‐2 cells (*P* < 0.05, Fig. 3A). SIRT6 knockdown notably suppressed migration of Saos‐2 and U2OS cells (*P* < 0.05 for both, Fig. 3B and Fig. S1A). Transwell assays explored that SIRT6 knockdown significantly reduced the migratory and invasive abilities of Saos‐2 and U2OS cells (*P* < 0.05 for both, Fig. 3C and Fig. S1B). In turn, SIRT6 overexpression was confirmed by immunoblotting in MG‐63 cells (*P* < 0.05, Fig. 3D). Subsequently, SIRT6 overexpression notably facilitated MG‐63 cell migration and invasion *in vitro* (*P* < 0.05 for both, Fig. 3E,F). Furthermore, our data indicated that modulating SIRT6 expression showed no significant effect on proliferation of OS cells (Fig. 3G). Thus, SIRT6 exerts a pro‐metastatic role in OS cells.

**Figure 3:** SIRT6 contributes to the migration and invasion of OS cells. (A) Saos‐2 cells that were transfected with scrambled siRNA (siNC) or siSIRT6 were confirmed by immunoblotting. *P < 0.05. (B) SIRT6 knockdown suppressed migration of Saos‐2 cells as suggested by wound healing assays. (C) Transwell assays confirmed that SIRT6 silencing prohibited migration and invasion in Saos‐2 cells. *P < 0.05. (D) MG‐63 cells that were transfected with control vector or pc‐DNA3.1‐SIRT6 were confirmed by immunoblotting. *P < 0.05. (E) SIRT6 restoration facilitated migration of MG‐63 cells. (F) Transwell assays confirmed that SIRT6 overexpression promoted migration and invasion in MG‐63 cells. *P < 0.05. (G) Modulating SIRT6 expression showed no significant effect on cell proliferation in both Saos‐2 and MG‐63 cells.

### SIRT6 regulates MMP9 abundance in OS cells

To disclose the potential molecular mechanisms involved in the role of SIRT6 in OS cells, we searched for candidate mediators of SIRT6 via a literature review. MMP9, a pro‐metastatic factor in human OS 24, 25, is up‐regulated by SIRT6 and promotes metastasis of NSCLC 21. Further experiments were performed to confirm that MMP9 is a potential downstream mediator of SIRT6 in OS. The levels of MMP9 protein between OS cell lines and NB tissues were detected by immunoblotting. The levels of MMP9 in all OS cell lines were significantly increased compared with NB tissues (*P* < 0.05 for all, Fig. 4A). The expression trend of MMP9 was similar to SIRT6 expression in OS cell lines. Interestingly, SIRT6 knockdown reduced the level of MMP9 protein in Saos‐2 cells (*P* < 0.05, Fig. 4A), while SIRT6 overexpression increased the level of MMP9 in MG‐63 cells (*P* < 0.05, Fig. 4B). We further explored whether MMP9 mediated the role of SIRT6 in OS cells. pcDNA3.1‐MMP9 was employed to disclose whether MMP9 restoration abolished the effects of SIRT6 knockdown on OS cells. As shown in Fig. 5A, pcDNA3.1‐MMP9 transfection significantly increased the level of MMP9 in SIRT6 down‐regulating Saos‐2 cells (*P* < 0.05). Consequently, MMP9 restoration promoted the metastatic behaviors of Saos‐2 cells with increased cell migration and invasion (*P* < 0.05 for both, Fig. 5B). SIRT6 overexpressing MG‐63 cells were transfected with MMP9 siRNA and scrambled siRNA (*P* < 0.05, Fig. 5C). MMP9 knockdown abolished the pro‐metastatic effects of SIRT6 on MG‐63 cells (*P* < 0.05, Fig. 5D). These experiments suggest that SIRT6 promotes the migration and invasion of OS cells possibly by up‐regulating MMP9.

**Figure 4:** SIRT6 positively regulates MMP9 abundance in OS cells. (A) The differences in the expression of MMP9 between four different OS cell lines (Saos‐2, MG‐63, U2OS and 143B) and NB specimens. *P < 0.05. (B) Saos‐2 cells that were transfected with scrambled siRNA (siNC) or siSIRT6 were confirmed by immunoblotting. SIRT6 knockdown down‐regulated the level of MMP9 in Saos‐2 cells. *P < 0.05. (C) MG‐63 cells that were transfected with control vector or pc‐DNA3.1‐SIRT6 were confirmed by immunoblotting. SIRT6 overexpression increased the level of MMP9 in MG‐63 cells. *P < 0.05.

**Figure 5:** MMP9 is a potential downstream mediator of SIRT6. (A) The level of MMP9 was down‐regulated by SIRT6 siRNA, while pcDNA3.1‐MMP9 transfection reversed the inhibitory effect of SIRT6 knockdown on MMP9 in Saos‐2 cells. *P < 0.05. (B) MMP9 restoration abrogated the effects of SIRT6 loss on Saos‐2 cells with increased cell migration and invasion *in vitro*. *P < 0.05. (C) SIRT6 overexpressing MG‐63 cells that were transfected with MMP9 siRNA and scrambled siRNA (siNC) were subjected to immunoblotting. *P < 0.05. (D) MMP9 knockdown abrogated the pro‐metastatic effects of SIRT6 on MG‐63 cells. *P < 0.05.

### The ERK1/2–MMP9 pathway may be involved in the role of SIRT6

As previous studies have identified that the mitogen‐activated protein kinase kinase (MEK)–ERK1/2 pathway regulates MMP9 expression and subsequently controls cancer cell migration and invasion 21, 26, we investigated whether the MEK–ERK1/2 pathway was involved in the role of SIRT6 in OS. Interestingly, we found that the levels of phosphorylated ERK1/2 and MMP9 were remarkably decreased after SIRT6 knockdown (Fig. 6A) in Saos‐2 cells. Consistently, SIRT6 overexpression increased the activation of the MEK–ERK1/2 pathway and MMP9 level in MG63 cells (Fig. 6B). Notably, PD098059 and PD0325901, inhibitors of MEK 27, 28, reduced the levels of phosphorylated ERK1/2 and blocked the promoting effect of SIRT6 on MMP9 abundance in MG‐63 cells (Fig. 6B,C). Moreover, PD098059 treatment reduced migration and invasion of SIRT6‐overexpressing MG‐63 cells (*P* < 0.05 for both; Fig. S2). Therefore, these results indicate that the ERK1/2–MMP9 pathway may be involved in the SIRT6‐induced OS progression.

**Figure 6:** SIRT6 regulates the activation of the ERK1/2–MMP9 pathway. (A) Saos‐2 cells that were transfected with scrambled siRNA (siNC) or siSIRT6 were confirmed by immunoblotting. SIRT6 knockdown decreased the levels of phosphorylated ERK1/2 and MMP9 in Saos‐2 cells. *P < 0.05. (B,C) MG‐63 cells that were transfected with control vector or pc‐DNA3.1‐SIRT6 were confirmed by immunoblotting. SIRT6 overexpression increased the levels of phosphorylated ERK1/2 and MMP9 in MG‐63 cells. SIRT6‐overexpressing MG‐63 cells were exposed to the specific inhibitors of MEK, PD098059 (50 μm) and PD0325901 (50 nm) for 30 min. Both PD098059 and PD0325901 blocked the activation of the ERK1/2–MMP9 pathway despite SIRT6 overexpression. *P < 0.05.

## Discussion

Sirtuin 6 is selectively down‐regulated in several human cancers 11. On the other hand, overexpression of SIRT6 is observed in HCC and NSCLC 15, 21. This evidence supports conflicting expressions for SIRT6 in cancer. In the present study, we demonstrated that SIRT6 was significantly overexpressed in OS tissues and cells. Recent studies revealed that the ubiquitin ligase and transcription factors are up‐regulators of SIRT6. Mammalian ubiquitin‐specific peptidase 10 deubiquitinates SIRT6 and protects it from proteasome‐mediated degradation in human colon cancer cells 29. Kim *et al*. 30 showed that SIRT1 forms a complex with forkhead box O3a and nuclear respiratory factor 1 on the SIRT6 promoter and positively regulates expression of SIRT6 in mice liver. Human males absent on the first is a histone acetyltransferase that can significantly increase the protein and mRNA levels of SIRT6 in HCC by binding to its promoter 31. Recently, Zhang *et al*. 32 reported that p53 directly activates the expression of SIRT6. The reason for differential SIRT6 expression in OS remains a challenge and requires further investigation.

Aberrant expression of SIRT6 has been considered as a novel biomarker for predicting prognosis of cancer patients 11, 13, 15, 21, 22. For instance, low expression levels of SIRT6 predict poor prognosis and reduced tumor‐free survival rates in several human cancers 11. Up‐regulation of SIRT6 was highly associated with shorter survival in HCC 15. A recent study showed that high SIRT6‐expressing NSCLC patients have a lower cumulative survival rate as compared with low SIRT6‐expressing patients 21. Moreover, the subcellular localization of SIRT6 is associated with poor prognosis of patients with NSCLC 22. Our study is the first to report that up‐regulation of SIRT6 correlated with clinicopathological features and poor prognosis of OS patients. This study has made an incremental contribution in the prognostic significance of SIRT6 in human cancer.

Tumor metastasis and recurrence are at the root of poor clinical outcome for OS patients 33. Meanwhile, tumor metastasis and recurrence are inseparable from enhanced cancer cell mobility. Our data revealed that SIRT6 promoted migration and invasion of OS cells without affecting cell proliferation, which is consistent with the role of SIRT6 in NSCLC 21. These results suggest that SIRT6 promotes tumor progression probably by exerting a pro‐metastatic role in OS. Tumor metastasis is a multistep process, and numerous studies have found that MMPs facilitate metastasis by degrading the extracellular matrix 34. MMP9, an important member of the zinc‐metalloproteinase family, promotes tumor metastasis via degradation of the extracellular matrix 35. MMP9 facilitates cancer cell migration and invasion by degrading the major extracellular matrix components type I and IV collagens in OS 36. MMP9 overexpression functions as a predictive marker for poor prognosis in patients with OS 37. The MMP9 gene promoter regions contain *cis*‐elements for the Sp1 transcription factor, and ERK activation is crucial for Sp1‐mediated MMP9 expression 38. The MEK–ERK1/2 pathway facilitates the metastasis of OS via its downstream targets 39, 40. Previous research has identified that MMP9 is a downstream target of the MEK–ERK1/2 pathway and subsequently controls cancer cell migration and invasion 21. SIRT6 promoted metastasis of NSCLC via the ERK/1/2–MMP9 pathway 21. Our present data revealed a link between SIRT6 overexpression and increased MMP9 level as well as increased ERK1/2 phosphorylation. MMP9 functioned in SIRT6‐induced OS cell migration and invasion. SIRT6‐mediated effects were MEK‐dependent, since MEK inhibitors (PD098059 and PD0325901) blocked the promoting effects of SIRT6 on ERK1/2 phosphorylation, MMP9 expression and mobility of OS cells, which is consistent with a previous report 36. These results suggest that the ERK1/2–MMP9 pathway may be involved in the SIRT6‐induced OS progression. Here, we explored the role of SIRT6 and its underlying mechanisms by modulating the SIRT6 level using siRNA and an expression plasmid, which is easy to achieve. SIRT6 has two major biochemical activities, functioning as a deacetylase and a mono‐ADP ribosyltransferase 41, 42. The important of SIRT6 activity has been confirmed in other studies 43, 44, 45. The important of SIRT6 activity in OS is a new challenge to be investigated in our further study.

In summary, we find that SIRT6 overexpression is commonly observed in OS. High expression of SIRT6 confers poor prognosis for OS patients. SIRT6 facilitates migration and invasion of OS cells through the ERK1/2–MMP9 pathway. SIRT6 may serve as a prognostic indicator and a potential therapeutic target in OS.

## Conclusions

Our study recognized SIRT6 as a novel biomarker for predicting poor prognosis of OS patients. Next, we found that SIRT6 promoted migration and invasion of OS cells *in vitro*. Furthermore, MMP9 was identified as a potential functional mediator of SIRT6 in OS cells. Notably, the ERK1/2–MMP9 pathway probably played an essential role in SIRT6‐induced migration and invasion of OS cells. Our current study only focused on SIRT6 protein level in total cell/tissue lysates and suggested that the proposed mechanism might depend on SIRT6 levels. Further studies are needed to investigate SIRT6 localization or its enzymatic function as a deacylase/ribosyltransferase in OS cells. Recent studies reveal that ubiquitin ligase, microRNAs and transcription factors are down‐regulators or up‐regulators of SIRT6. The reason for differential SIRT6 expression in OS remains a challenge and requires further investigation.

## Author contributions

HL, ZZ and YT carried out the cell biology and molecular biology experiments, participated in the sequence alignment and drafted the manuscript. HL and YH participated in the design of the study and performed the statistical analysis. YH conceived of the study, and participated in its design and coordination and helped to draft the manuscript. All authors read and approved the final manuscript.

## Supporting information


**Fig. S1**. SIRT6 knockdown inhibits migration and invasion of U2OS cells.
**Fig. S2**. MEK inhibitor PD098059 abolished the pro‐metastatic effect of SIRT6 in MG‐63 cells.
